The article "Scolopendra subspinipes mutilans L. Koch Ameliorates Rheumatic Heart Disease by Affecting Relative Percentages of CD4+CD25+FoxP3 Treg and CD4+IL17 T Cells" was retracted in 2021. Reasons: errors in the materials; errors in the data; errors in the analysis; unreliable results or conclusions.

# *Scolopendra subspinipes mutilans L. Koch* Ameliorates Rheumatic Heart Disease by Affecting Relative Percentages of CD4^+^CD25^+^FoxP3 Treg and CD4^+^IL17 T Cells

**DOI:** 10.1155/2019/4674190

**Published:** 2019-07-14

**Authors:** Tiechao Jiang, Qini Zhao, Hongyan Sun, Lirong Zhang, Shanshan Song, Hongli Chi, Hui Zhou

**Affiliations:** ^1^Department of Cardiovascular Medicine, China-Japan Union Hospital of Jilin University, Changchun 130033, China; ^2^Jilin Provincial Precision Medicine Key Laboratory for Cardiovascular Genetic Diagnosis, Changchun 130033, China; ^3^Department of Pathology, China-Japan Union Hospital of Jilin University, Changchun 130033, China; ^4^Department of Radiology, College of Public Health, Jilin University, Changchun 130021, China; ^5^Department of EICU, The First Hospital of Jilin University, Changchun 130021, China; ^6^Department of Anesthesiology, China-Japan Union Hospital of Jilin University, Changchun 130033, China

## Abstract

(*Scolopendra subspinipes mutilans L. Koch*. (SSLK) helps reduce the risk of coronary heart disease (CHD) but its effects on rheumatic heart disease (RHD) patients remain unclear. 80 RHD patients were recruited and randomly assigned into SG (to receive SSLK treatment) and CG (to receive placebo) groups, and the intervention lasted for 3 months. The following cardiac indexes were measured, including mean arterial pressure (MAP), heart rate (HR), central venous pressure (CVP), blood lactate, fatigue, shortness of breath, palpitation, and chest pain. ELISA kits were used to analyze creatine kinase isoenzyme (CK-MB), serum troponin T (cTnT), CRP, IL-1*β*, IL-6, and TNF-*α*, malondialdehyde (MDA), and superoxide dismutase (SOD). Relative percentages of CD4^+^CD25^+^FoxP3 regulatory (Treg) and CD4^+^IL-17 T cells were measured using flow cytometry. After 3-month therapy, SSLK intervention improved MAP, HR, CVP, fatigue, palpitation, and shortness breath of CHD patients, reduced the levels of blood lactate, CK-MB, cTnT, CRP, IL-1*β*, IL-6, TNF-*α*, MDA, and increased SOD level (*p* < 0.05). Meanwhile, SSLK treatment increased the percentages of CD4^+^CD25^+^FoxP3 Treg cells and reduced relative percentages of CD4^+^IL-17 T cells in a dose-dependent way (*p* < 0.05). Relative percentage of CD4^+^CD25^+^FoxP3 Treg cells had negative relationship while CD4^+^IL17 T cells had positive relationship with CK-MB, cTnT, CRP, and TNF-a (*p* < 0.01). SSLK ameliorated RHD by affecting the balance of CD4^+^CD25^+^FoxP3 Treg and CD4^+^IL17 T cells.

## 1. Introduction

Rheumatic heart disease (RHD) is a sequel of acute rheumatic fever (ARF) [1, 2] and an autoimmune disease caused by the damage to heart valves [3] or hemolytic streptococcal infection [4]. According to statistics, there are more than 15.6 million RHD patients in the world [5]. The prevention and treatment of RHD is still a common public health issue and causes a global burden. Antibiotics are often used in the treatment of RHD to prevent infection and the inflammation of the heart and other symptoms [6, 7]. However, a frequent and distressing complication often occurs after the treatment. Some pathogen can develop antibiotic resistance and make the treatment ineffective [8]. Furthermore, antibiotics produce toxicity [9] and cause drug-drug interaction [10], which will further contribute to RHD progression. It is highly needed to explore new effective medicine with fewer side effects.

*Scolopendra subspinipes mutilans L. Koch *(SSLK), ancient antipyretic traditional Chinese medicine, can improve blood circulation, relieve blood stasis [11], and prevent heart failure by attenuating postinfarct remodeling [12]. SSLK has been reported to control vascular disease via its anti-inflammatory activities [13]. SSLK can reduce the risk of heart disease by improving the biochemical indices of patients [14]. More work indicates that SSLK can regulate fatty acids metabolism by exerting antiadipogenic activity via the inhibition of the expression of C/EBP*β*, C/EBP*α*, and PPAR*γ* and the Akt signaling pathway in adipocytes [15].

It has been reported that CD4^+^T cells are the major effector cells in the heart valve of RHD patients, and the number of these cells is increased in the peripheral blood of RHD patients [16]. There are approximately 5% to 10% of CD4^+^T cells in peripheral blood and spleen tissues of healthy persons. CD25, TGF-beta, and forkhead box protein P3 (FoxP3) are highly expressed in T cells [17]. These proteins play crucial roles in the immunosuppressive functions of regulatory T (Treg) cells [18]. CD4^+^CD25^+^Treg cells are generated in the thymus and have been reported to mitigate autoimmune myocarditis [19]. The dysfunction of CD4^+^CD25^+^Treg cells may lead to RHD occurrence and FoxP3 regulates Treg cell development and function [20, 21]. CD4^+^IL-17 T cells have been reported to be associated with bacterial infection and inflammatory responses [22, 23].

SSLK reduces the risk of coronary heart disease (CHD) [24]. However, the effects of SSLK on RHD remain unknown and related molecular mechanisms are unclear. High-level Th17/Treg ratio has been found to be associated with the risk and progression of RHD [25]. CD4^+^IL17 T cells are the main Th17 cell subsets [26] and CD4^+^CD25^+^FoxP3 Treg cells are the main Treg cell subsets [27]. Thus, SSLK may exert beneficial effects on RHD patients by affecting the levels of CD4^+^CD25^+^FoxP3 Treg and CD4^+^IL17 T cells. Therefore, in this study, peripheral blood samples were collected from RHD patients to investigate the effects of SSLK on regulatory T lymphocytes. To investigate the changes of relative percentages of CD4^+^CD25^+^Treg and CD4^+^IL-17 T cells induced by SSLK, the study may provide new molecular mechanism for RHD treatment.

## 2. Materials and Methods

### 2.1. Materials

FITC mouse anti-human CD4 (Clone RPA-T4), an isotype control mouse IgG1-FITC (Clone MOPC-21), APC mouse anti-human CD25 (Clone M-A251), an isotype control anti-APC mouse IgG1 (Clone MOPC-21), PE Mouse anti-Human FoxP3 (Clone 259D/C7), and an isotype control PE mouse IgG1 (Clone MOPC-21) were purchased from BD eBioscience (BD Bioscience, San Jose, CA, USA). Ficoll-Paque was purchased from Sigma (Louis, MO, USA). M-MLV First Strand Kit was purchased from Invitrogen (Shanghai, China). Power SYBR Green PCR Master Mix was purchased from ABI (Foster, CA, USA).

### 2.2. Participants

The study was approved by the Human Research Ethics Committee of China-Japan Union Hospital of Jilin University (Changchun, China, approval no. 2015NXY) and all participants signed informed consent. From November 2015 to July 2016, 227 CHD patients were recruited at our hospital. All patients were diagnosed with RHD based on clinical symptoms, rheumatic fever history, and cardiac ultrasonography.

### 2.3. Inclusion Criteria

All patients were diagnosed with rheumatic mitral valve disease by medical history, physical examination, laboratory examination, echocardiography, and surgery.

### 2.4. Exclusion Criteria

The patients would be excluded if they had the following symptoms: acute myocardial infarction and severe heart failure; psychiatric abnormalities and being unable to correctly describe their symptoms and other autoimmune system diseases (such as rheumatoid arthritis); or systemic lupus erythematosus.

### 2.5. Patient Grouping

After applying inclusion criteria and exclusion criteria, a total of 80 RHD patients entered the present study at China-Japan Union Hospital of Jilin University. SSLKs were purchased from Beijing Tongrentang Pharmacy (Beijing, Chin) to make fine powder. The patients were evenly and randomly assigned into two groups: SSLK (SG, orally given 100-mg SSLK powder every morning) and control (CG, orally given 100-mg placebo every morning). The whole duration of the treatment was three months. Liver function was measured using liver function monitoring system (LiMON Leberfunktionsmonitor, Pulsion Medical Systems AG, Munich, Germany). Renal function was measured using blood urea nitrogen, serum creatinine, and estimated glomerular filtration rate according to previous reports [28]. Meanwhile, side effects (dry mouth, diarrhea, dizziness, weakness, no appetite or nausea, headache, fatigue, nightmares, and so on) were measured according to self-reported physical activity.

### 2.6. Hemodynamics and Arterial Blood Gas Index

Dopamine would be considered when the severe condition of RHD occurred. Mean arterial pressure (MAP), heart rate (HR), central venous pressure (CVP, evaluated by ultrasound of the internal jugular vein), partial pressure of oxygen (PaO_2_), and blood lactate levels were measured at 0 months, 1 month, 2 months, and 3 months.

### 2.7. Serum Levels of Inflammatory Cytokines

The serum concentrations of C-reactive protein (CRP, Cat. No. ab136176), tumor necrosis factor-a (TNF-a, Cat. No. ab9348), IL-1*β* (Cat. No. ab46052), IL-6 (Cat. No. ab178013), IL-10 (Cat. No. ab46034), and TGF-*β* (Cat. No. ab100647) were measured using the ELISA kits from Abcam (Shanghai, China).

### 2.8. Cardiac Biomarker Levels

After 0-, 1-, 2- and 3-month treatment, the creatine kinase isoenzyme (CK-MB), serum cardiac troponin T (cTnT), malondialdehyde (MDA), and superoxide dismutase (SOD) were detected by an automatic biochemical analyzer (Hitachi 7600P, Hitachi, Japan).

### 2.9. The Measurement of CD4^+^CD25^+^FoxP3 Treg and CD4^+^IL-17 T Cells

Five-mL venous blood was taken aseptically from each subject at 0 months and 3 months and heparinized anticoagulated. The blood samples were processed within 2 h. Five-mL venous blood and equal volume of sterile saline were used to dilute the venous blood and mixed thoroughly to extract peripheral blood mononuclear cells (PBMCs). PBMCs were prepared using Ficoll-Paque density gradient centrifugation. CD4^+^ cells were gated on forward and side scatter for lymphocyte purity in the gate. Relative percentages of CD4^+^CD25^+^FoxP3 Treg and CD4^+^IL-17 T cells were analyzed by flow cytometry.

### 2.10. The Effects of SSLK on Relative Percentages of CD4^+^CD25^+^FoxP3 Treg and CD4^+^IL-17 T Cells

Above PBMCs were cultured in DMEM medium with fetal bovine serum (Cat. No. TM999) to a final concentration of 10% and penicillin/streptomycin at 1%. The cells were adjusted to a density of 1 × 10^5^ cells/mL, added to a 96-cell plate (100 *μ*L/per cell), and cultured at 95% air, 5% CO_2_, and 37°C. SSLK powder was added to the medium with final concentration from 0 to 10 *μ*g/mL. After 48 h, PBMCs were stained by surface marker CD4 and CD25 antibodies firstly. After fixation and permeabilization, PBMCs were then stained by Foxp3 and IL-17 antibodies. Relative percentages of CD4^+^CD25^+^FoxP3 Treg and CD4^+^IL-17 T cells were analyzed by flow cytometry.

### 2.11. Statistical Analysis

SPSS18.0 statistical software was used for data analysis. Quantitative variables were expressed as mean values ± S.D. (standard derivative). Independent samples T-test and one-way analysis of variance (ANOVA) were used to compare the data difference between CG and SG groups. Chi-square test was used to compare the number difference between two groups. The correlation between two variables was analyzed using Pearson correlation coefficient test.* p* < 0.05 indicates the difference was statistically significant.

## 3. Results

### 3.1. Clinical Characteristics

The baseline clinical characteristics of RHD patients from two groups were shown in Table 1. There was no significant difference in age, body mass index, triglyceride, total cholesterol, low density lipoprotein cholesterol, and high-density lipoprotein cholesterol between the two groups (*p* > 0.05). At the same time, there were more female patients in the case group.

### 3.2. SSLK Consumption Improved the Complications of CHD Patients

The statistical difference for the cases of fatigue, chest pain, palpitation, and short breathing was insignificant between the CG and SG groups (Table 2,* p* > 0.05). After 3-month therapy, the symptoms were improved in SG when compared with CG group except chest pain (Table 2,* p* < 0.05). SSLK treatment improved the complications of CHD patients.

### 3.3. SSLK Treatment Reduced the Level of Blood Lactate

The statistical differences for the levels of MAP, HR, CVP, arterial PaO2, and blood lactate content were insignificant between two groups at 0 months and 1 month (Table 3,* p* > 0.05); MAP, HR, CVP, Pao2, and blood lactate content in the SG were lower than in the CG group after 2 months (Table 3,* p* < 0.05). The results suggested that SSLK treatment could not affect MAP, HR, CVP, PaO_2_, and blood lactate in a short term.

### 3.4. SSLK Treatment Reduced the Inflammatory Cytokines Levels

The statistical differences for the levels of CRP, TNF-a, IL-1*β*, and IL-6 levels were insignificant between the two groups at 0 months (Table 4,* p* > 0.05). The concentrations of CRP, TNF-a, IL-1*β*, and IL-6 in the SG group were lower than in the CG group (Table 4,* p* < 0.05). The results suggested that SSLK reduced the inflammatory cytokines levels.

### 3.5. SSLK Treatment Improved Myocardial Enzyme Levels

The statistical differences of CK-MB, cTnT, MDA, and SOD levels were insignificant between the two groups (P<0.05, Table 3). The concentrations of CK-MB, cTnT, and MDA in the SG group were lower than in the CG group while SOD had reverse results (Table 5,* p *< 0.05). The results suggested that SSLK treatment improved myocardial enzyme levels.

### 3.6. SSLK Treatment Improved Serum Levels of Inflammatory Factors

ELISA analysis showed that SSLK treatment reduced the serum levels of IL-1*β* (Figure 1(a)) and IL-6 (Figure 1(b)) and increased the levels of IL-10 (Figure 1(c)) and TGF-*β* (Figure 1(d)) when compared with the CG group (*p* < 0.05). SSLK treatment improved serum levels of inflammatory factors.

### 3.7. SSLK Treatment Affected Relative Percentages of CD4^+^CD25^+^FoxP3 Treg and CD4^+^IL-17 T Cells in PBMCs

Before SSLK intervention, the average percentages of CD4^+^CD25^+^FoxP3 Treg cells (Figure 2(a)) and CD4^+^IL-17 T cells (Figure 2(b)) were 3.5% and 7.2% in CG group, respectively. The average percentages of CD4^+^CD25^+^FoxP3 Treg cells (Figure 2(c)) and CD4^+^IL-17 cells (Figure 2(d)) were 3.7% and 6.9%. The statistical differences for the percentages of CD4^+^CD25^+^FoxP3 Treg cells and CD4^+^IL-17 T cells were insignificant (*p* > 0.05). After 3-month SSLK intervention, the average percentages of CD4^+^CD25^+^FoxP3 Treg cells (Figure 2(e)) and CD4^+^IL-17 T cells (Figure 2(f)) were 3.2% and 6.5% in CG group, respectively. The average percentages of CD4^+^CD25^+^FoxP3 Treg cells (Figure 2(g)) and CD4^+^IL-17 cells (Figure 2(h)) were 5.8% and 3.4% in the SG group, respectively. SSLK treatment increased the percentages of CD4^+^CD25^+^FoxP3 Treg cells (from 3.2 ± 0.5 to 5.8 ± 0.7) and reduced the percentages of CD4^+^IL-17 T cells (from 6.5 ± 0.9 to 3.4 ± 0.6). The results suggested that SSLK consumption affected the percentages of CD4^+^CD25^+^FoxP3 Treg cells and CD4^+^IL-17 T cells in PBMCs.

### 3.8. The Effects of SSLK on the Percentage of CD4^+^CD25^+^FoxP3 Treg and CD4^+^IL-17 T Cells in PBMCs

Figure 3 showed that SSLK increased the percentage of CD4^+^CD25^+^FoxP3 Treg cells (Figure 3(a)) and reduced the percentage of CD4^+^IL-17 T cells (Figure 3(b)) in a dose-dependent way in PBMCs. The results showed that SSLK intervention regulated the percentages of CD4^+^CD25^+^FoxP3 Treg and CD4^+^IL-17 T cells in PBMCs.

### 3.9. The Percentage of CD4^+^CD25^+^FoxP3 Treg Cells Had Negative Relationship with CK-MB, cTnT, CRP, and TNF-a

Pearson correlation coefficient test showed that, with the increase in the percentage of CD4^+^CD25^+^FoxP3 Treg cells, the levels of CK-MB (Figure 4(a)), cTn1 (Figure 4(b)), CRP (Figure 4(c)), and TNF-a (Figure 4(d)) were reduced. The percentage of CD4^+^CD25^+^FoxP3 Treg cells had negative relationship with the levels of CK-MB, cTnT, CRP, and TNF-a since rho < -0.5 and* p* < 0.01.

### 3.10. The Percentage of CD4^+^IL-17 T Cells Had Positive Relationship with CK-MB, cTnT, CRP, and TNF-a

Pearson correlation coefficient test showed that, with the increase in the percentage of CD4^+^IL-17 T cells, the levels of CK-MB (Figure 5(a)), cTn1 (Figure 5(b)), CRP (Figure 5(c)), and TNF-a (Figure 5(d)) were increased. The percentage of CD4^+^IL-17 T cells had positive relationship with the levels of CK-MB, cTnT, CRP, and TNF-a since rho > 0.5 and* p* < 0.01.

## 4. Discussion

SSLK reduced the levels of cardiac biomarkers (CK-MB and cTnT) and inflammatory cytokines in RHD patients (Table 4 and Figure 1), suggesting it can regulate inflammatory activity of patients. The reduction of CD4^+^CD25^+^FoxP3 Treg cells and the increase in CD4^+^IL-17 cells in PBMCs may be associated with poor prognosis of RHD. CD4^+^CD25^+^Tregs [29] and CD4^+^CD25^+^FoxP3 Treg cells [30] regulated the immune activity in heart disease. Relative percentages of CD4^+^CD25^+^Tregs and CD4^+^CD25^+^FoxP3 Treg cells in PBMCs in the SG group were higher than in the CG group (Figure 2, P<0.05). SSLK has antibacterial [31], anticoagulant [32], and anti-inflammatory [33] properties. SSLK intervention may improve CHD symptoms of the patients by increasing the percentage of CD4^+^CD25^+^FoxP3 Treg cells and reducing the percentage of CD4^+^IL-17 cells in PBMCs and maintained their balance (Figure 6). The immunomodulatory function of Treg cells is also closely related to the secretion of cytokines in peripheral blood plasma. IL-10 and TGF-*β* are secreted by Treg T cells, control inflammation, and regulate immunosuppression [34, 35]. In addition, TGF-*β*1 can induce the FoxP3 gene expression, participate in the accurate differentiation of Treg cells, and promote the survival of natural Treg cells [36]. Previous studies have demonstrated that TGF-*β*, which bind to cell membranes, increased the number of CD4^+^CD25^+^Treg cells and also affected Treg function [37, 38]. SSLK intervention increased the serum levels of IL-10 and TGF-*β* in RHD patients (Figures 1(c) and 1(d)). A decrease in the secretion of IL-10 and TGF-*β* in the serum of RHD patients may affect the number of Treg cells and impair their functions. IL-10 polymorphism has been found to be associated with progression of RF/RHD, suggesting its important role in controlling CHD risk [39]. SSLK treatment reduced the levels of IL-1 *β* and IL-6 and effectively controlled inflammation responses.

There is significant deficiency of Tregs (CD4^+^CD25(med-high)CD127(low) Foxp3(high)) in patients of chronic RHD [40] while increased percentage of Th17 cell-associated cytokines plays crucial roles in the progression of RHD [41]. The present work showed that SSLK treatment increased the percentages of CD4^+^CD25^+^FoxP3 Treg cells and reduced the percentages of CD4^+^IL-17 T cells in a dose-dependent way (*p* < 0.05). The percentage of CD4^+^CD25^+^FoxP3 Treg cells had negative relationship with CK-MB, cTnT, CRP, and TNF-a (Figure 4). The percentage of CD4^+^IL-17 T cells had positive relationship with CK-MB, cTnT, CRP, and TNF-a (Figure 5). CK-MB and cTnT are the important cardiac biomarkers associated with RHD risk [42]. CRP [43] and TNF-a [44] are related to the inflammation of CHD. Thus, SSLK ameliorated RHD by affecting CD4^+^CD25^+^FoxP3 Treg and CD4^+^IL17 T cells.

Notably, to reduce inflammation, low-dose aspirin (50 mg/daily) was orally administrated in both group [45]. Although aspirin has been reported to increase the numbers of Treg cells, its effects on the control group were not found when compared with before treatment [46]. On the other hand, in the present study, the normal percentages of Treg and Th17 cells were not found in CHD patients, which may be caused by the small size (40 subjects in each group). The effects of SSLK on the CHD patients with normal percentages of CD4^+^CD25^+^FoxP3 Treg and CD4^+^IL-17 cells remain unclear. However, according to another report, the normal percentage of Treg cells should be existing even in severe gastrointestinal inflammation [47]. Much work needs to address these important issues in the future.

The cases of fatigue, chest pain, palpitation, and short breathing are the common complications of RHD. In the present study, the symptoms of fatigue and palpitation were all improved after SSLK intervention (Table 2, p < 0.05). Adverse reaction of SSLK was also analyzed, 2 patients had dizziness, weakness (1 case), and headache (1 case), and there were no liver, or kidney dysfunction, and/or other clinical abnormalities in the SSLK group. Notably, a SSLK treatment duration was 3 months. Traditional Chinese medicine is quite different with normal drug and cannot exert its function in human body immediately, and several months will be considered [48].

There are some limitations to the present work. The subsequent clinical characteristics were not investigated further after stopping taking SSLK. In addition, CD4^+^CD25^+^Treg cells was only detected in PBMCs from peripheral blood, and our results would be affected by the fact that Treg cells were a small fraction in RHD patients. An additional marker FoxP3 was used to distinguish between functional Treg cells and immature nonfunctional Treg cells. Therefore, further study should be performed to observe FOXP3 gene expression in the CD4^+^CD25^+^ Treg cells. The epigenetic regulation of CD4^+^CD25^+^Treg cells is closely related to human heart diseases. Therefore, it is very important to evaluate the epigenetic regulation of FoxP3 gene in RHD patients. The small sample size of this study should be further expanded to a larger population of RHD patients and follow-up period should be longer in order to gain the key advantages of SSLK. In Figure 1(d), the treatment seems to induce a separation for TGF-*β* between two different patient populations in the SG group (the median cuts sharply between two groups of red dots). The problem may be caused by small population size. To address these issues, further work is highly demanded in the future.

## 5. Conclusions

SSLK treatment improved MAP, HR, CVP, fatigue, palpitation, and shortness breath in the CHD patients. Meanwhile, SSLK intervention reduced the levels of blood lactate, CK-MB, cTnT, CRP, IL-1*β*, IL-6, TNF-*α*, and MDA and increased SOD level. SSLK treatment reduced the levels of IL-1*β* and IL-6 and increased the levels of IL-10 and TGF-*β*. SSLK had better anti-inflammatory effects. No increased risk of serious adverse reactions such as bleeding was found. SSLK treatment increased the percentage of CD4^+^CD25^+^FoxP3 Treg cells and reduced the percentage of CD4^+^IL-17 T cells. SSLK ameliorated RHD by affecting the percentage of CD4^+^CD25^+^FoxP3 Treg and CD4^+^IL17 T cells.

## Figures and Tables

**Figure 1:** ELISA analysis of the effects of SSLK on the levels of cytokines and transcription factor. (a), the effects of SSLK on serum levels of IL-1*β*. (b), the effects of SSLK on serum levels of IL-6. (c), the effects of SSLK on serum levels of IL-10. (d), the effects of SSLK on the levels of TGF-*β*. In the SG group, the patients took SSLK and in the CG group, the patients took placebo (n = 40 for each group).*∗p* < 0.05 via a control group.

**Figure 2:** Flow cytometry analysis of the percentage of CD4^+^CD25^+^FoxP3 Treg and CD4^+^IL-17 T cells in PBMCs. (a), the percentage of CD4^+^CD25^+^FoxP3 Treg cells in the CG group before placebo intervention. (b), the percentage of CD4+IL-17 T cells in the CG group before placebo intervention. (c), the percentage of CD4^+^CD25^+^ FoxP3 Treg cells in the SG group before SSLK intervention. (d), the percentage of CD4^+^IL-17 T cells in the SG group before SSLK intervention. (e), the percentage of CD4^+^CD25^+^FoxP3 Treg cells in the CG group after 3-month placebo intervention. (b), the percentage of CD4+IL-17 T cells in the CG group after 3-month placebo intervention. (c), the percentage of CD4^+^CD25^+^ FoxP3 Treg cells in the SG group after 3-month SSLK intervention. (d), the percentage of CD4^+^IL-17 T cells in the SG group after 3-month SSLK intervention. In the SG group, the patients took SSLK and in the CG group, the patients took placebo.

**Figure 3:** The effects of SSLK on the percentage of CD4^+^CD25^+^FoxP3 Tregs and CD4^+^IL-17 T cells in PBMCs. (a), The effects of SSLK on the percentage of CD4^+^IL-17 T cells in PBMCs. (b), the effects of SSLK on the percentage of CD4^+^CD25^+^FoxP3 Treg cells in PBMCs. *∗p* <0.05 and *∗∗p* <0.01 via the 0-*μ*g/ml group.

**Figure 4:** The relationship between the percentage of CD4^+^CD25^+^FoxP3 Tregs and CK-MB,cTn1, CRP and TNF-*α*. (a), the relationship between the percentage of CD4^+^CD25^+^FoxP3 Tregs and CK-MB. (b), the relationship between the percentage of CD4^+^CD25^+^FoxP3 Tregs and cTn1. (c), the relationship between the percentage of CD4^+^CD25^+^FoxP3 Tregs and CRP. (d), the relationship between the percentage of CD4^+^CD25^+^FoxP3 Tregs and TNF-*α*. There was a strong negative relationship between two variables if rho values < -0.5.

**Figure 5:** The relationship between the percentage of CD4^+^IL-17 T cells and CK-MB,cTn1, CRP, and TNF-*α*. (a), the relationship between the percentage of CD4^+^IL-17 T cells and CK-MB. (b), the relationship between the percentage of CD4^+^IL-17 T cells and cTn1. (c), the relationship between the percentage of CD4^+^IL-17 T cells and CRP. (d), the relationship between the percentage of CD4^+^IL-17 T cells and TNF-*α*. There was a strong negative relationship between two variables if rho values > 0.5.

**Figure 6:** Schematic diagram of the effects of SSLK on CHD patients.

**Table 1:** Clinical characteristics of all participants.

	SSLK group (N=40)	Control group (N=40)	t/*χ*2 values	P values
Age, (years)	47.85 ± 9.95	45.20 ± 9.99	0.984	0.324
Female, n (%)	31(77.5)	28(70)	0.581	0.446
BMI, kg/m^2^	23.92 ± 2.26	23.32 ± 2.47	0.157	0.873
Smoking, n (%)	8 (20)	4 (10)	1.569	0.210
Diabetes, n (%)	5 (12.5)	6(15)	0.105	0.745
Hypertension, n (%)	32(78)	33(82.5)	0.082	0.775
Ongoing treatment				
Digoxin, n (%)	10(25)	8(20)	0.287	0.592
Aspirin, n (%)	22(55)	23(57.5)	0.051	0.822
NYHA classification				
II, n (%)	34(85)	35(87.5)	0.626	0.731
III, n (%)	6(15)	8(20)		
AF, n (%)	38(95)	33(82.5)		
Mitral stenosis,				
Moderate, n (%)	20(50)	23(57.5)	0.188	0.664
Severe, n (%)	15(37.5)	14(35)		
Aortic stenosis,				
Moderate, n (%)	3(7.5)	4(10)		
Severe, n (%)	2(5)	3(7.5)		
Tricuspid incompetence				
Mild, n (%)	28(70)	29(72.5)	0.583	0.747
Moderate, n (%)	6(15)	8(20)		
Severe, n (%)	2(5)	1(2.5)		
Plasma measurements,				
Triglycerides,	2.16 ± 1.24	1.94 ± 1.77	0.763	0.482
Total cholesterol (mmol/L),	5.33 ± 1.36	4.67 ± 1.41	1.639	0.163
LDL-C (mmol/L),	3.31 ± 0.89	3.46 ± 0.99	0.652	0.561
HDL-C (mmol/L),	1.59 ± 0.67	1.68 ± 0.39	0.758	0.478

Note: *SSLK, Scolopendra subspinipes mutilans L. Koch.* BMI, body mass index. NYHA, the New York Heart Association; AF, atrial fibrillation; LDL-C, low-density lipoprotein cholesterol; HDL-C, high-density lipoprotein cholesterol.

**Table 2:** The complications of rheumatic heart disease (RHD) patients between two groups.

Parameters	CG	SG	*p* values
0 months			
Fatigue, cases	35	33	0.531
Palpitation, cases	30	31	0.793
Dyspnea, cases	29	27	0.626
Chest pain grades, cases			
0	0	0	1.000
1	4	3	
2	5	7	
3	9	8	
4	8	7	
5	6	4	
6	5	6	
7	2	3	
8	1	2	
9	0	0	
10	10	0	
3 months			
Fatigue, cases	36	19	0.001
Palpitation, cases	30	21	0.036
Dyspnea, cases	28	16	0.007
Chest pain grades, cases			
0	3	8	0.935
1	6	10	
2	9	7	
3	8	5	
4	6	2	
5	5	3	
6	1	3	
7	2	1	
8	0	0	
9	0	0	
10	0	0	

Note: The pain grade scores (0-10) were analyzed and higher pain grades with higher scores were associated with more serious pain. The significant difference was analyzed by using a Chi-square test or one-way ANOVA. SG, SSLK group and CG, control group. There was significant difference if *p* < 0.05 vs. a control group.

**Table 3:** Comparison of hemodynamic parameters and arterial blood gas between two groups.

Parameters		0 months	1 month	2 months	3 months
MAP/mmHg	CG	73.65 ± 4.16	77.49 ± 6.23	78.21 ± 6.48	78.92 ± 7.25
	SG	75.12 ± 3.85	73.20 ± 5.76	70.33 ± 7.16	70.93 ± 7.64
F		0.245	0.268	2.495	2.996
*p* values		0.687	0.612	0.035	0.027
HR (times/min)	CG	76.48 ± 13.54	81.26 ± 15.37	80.38 ± 15.89	81.32 ± 15.71
	SG	77.62 ± 12.36	76.34 ± 9.18	70.96 ± 12.53	70.13 ± 13.99
F		0.109	0.436	3.168	3.656
*p* values		0.853	0.375	0.039	0.024
CVP/cmH_2_O	CG	15.41 ± 2.12	13.42 ± 3.84	14.61 ± 4.23	14.58 ± 4.35
	SG	15.65 ± 2.05	11.95 ± 4.13	10.36 ± 4.38	9.87 ± 4.69
F		0.063	1.169	4.219	5.324
*p* values		0.869	0.082	0.012	0.003
PaO_2_/mmHg	CG	156.26 ± 62.35	138.52 ± 40.24	130.44 ± 42.19	134.48 ± 43.01
	SG	168.23 ± 59.35	130.78 ± 35.17	111.36 ± 40.14	114.53 ± 42.38
F		0.246	0.835	3.237	3.064
*p* values		0.627	0.102	0.027	0.031
Blood lactate /mmol/L	CG	0.47 ± 0.10	0.85 ± 0.26	1.36 ± 0.36	1.34 ± 0.21
	SG	0.51 ± 0.16	0.73 ± 0.39	1.21 ± 0.30	1.22 ± 0.33
F		0.878	1.943	2.053	2.246
*p* values		0.126	0.051	0.042	0.039

Note: MAP, mean arterial pressure; HR, heart rate; CVP, central venous pressure and PaO2, Partial Pressure of Oxygen. SG, SSLK group and CG, control group. There was significant difference if *p* < 0.05 vs. a control group.

**Table 4:** The concentrations of CRP, TNF- a, IL-1, and IL-6 between two groups.

Parameters		0 months	1 month	2 months	3 months
CRP (*μ*g/mL)	CG	9.81 ± 1.32	79.36 ± 8.57	76.15 ± 9.25	56.23 ± 5.26
	SG	10.12 ± 1.26	62.21 ± 6.29	45.62 ± 3.26	39.58 ± 3.54
F		0.563	2.140	14.363	12.072
*p* values		0.451	0.022	0.001	0.001
TNF-*α* (pg/mL)	CG	11.32 ± 3.24	45.31 ± 5.26	24.15 ± 5.05	22.23 ± 4.25
	SG	10.29 ± 3.18	34.18 ± 2.95	18.23 ± 3.12	12.68 ± 2.52
F		1.027	9.741	13.981	15.327
*p* values		0.068	0.003	0.002	0.001
IL-6/(ng/L)	CG	21.15 ± 3.26	53.62 ± 11.05	68.29 ± 10.26	35.21 ± 9.26
	SG	20.59 ± 3.52	34.26 ± 5.62	23.46 ± 3.52	17.62 ± 4.76
F		0.217	12.451	22.461	38.972
*p* values		0.822	0.001	0.001	0.001
IL-1/(ng/L)	CG	18.26 ± 4.26	67.59 ± 8.26	59.26 ± 7.52	43.26 ± 5.21
	SG	18.15 ± 4.31	53.26 ± 6.05	31.25 ± 6.20	21.36 ± 4.74
F		0.116	8.642	12.673	36.519
*p* values		0.824	0.003	0.001	0.001

Note: CRP, C-creative protein; TNF-a, tumor necrosis factor; IL-1, interleukin-1 and IL-6, interleukin-6. SG, SSLK group and CG, control group. There was significant difference if *p* < 0.05 vs. a control group.

**Table 5:** Comparison of cardiac marker between two groups.

Parameters		0 months	1 month	2 months	3 months
CK-MB/	CG	7.61 ± 1.52	41.35 ± 12.20	52.26 ± 13.36	33.65 ± 8.26
(ng/mL)	SG	7.26 ± 1.46	26.58 ± 10.54	34.69 ± 11.25	21.26 ± 7.26
F		0.098	32.147	22.654	18.761
*p* values		0.912	0.001	0.001	0.001
cTnl/(ng/mL)	CG	0.01 ± 0.01	0.61 ± 0.23	1.38 ± 0.51	0.84 ± 0.35
	SG	0.01 ± 0.01	0.41 ± 0.28	0.76 ± 0.21	0.28 ± 0.12
F		0	16.423	25.349	45.678
*p* values		1.000	0.002	0.001	0.001
MDA/	CG	3.51 ± 0.89	7.68 ± 0.65	7.34 ± 0.58	6.84 ± 0.48
(nmol/mL)	SG	3.48 ± 0.79	5.87 ± 0.79	5.74 ± 0.83	4.26 ± 0.36
F		0.082	9.856	10.154	15.483
*p* values		0.947	0.002	0.002	0.001
SOD/	CG	120.35 ± 18.26	66.82 ± 17.65	78.52 ± 23.15	84.51 ± 26.03
(UN/mL)	SG	119.45 ± 17.36	88.26 ± 13.62	95.62 ± 24.58	108.26 ± 25.15
F		0.085	14.872	16.485	20.163
*p* values		0.793	0.002	0.001	0.001

Note: CK-MB, creatine kinase isoenzyme; cTnT, cardiac troponin T; MDA, malondialdehyde and SOD, superoxide dismutase. SG, SSLK group and CG, control group. There was significant difference if *p* < 0.05 vs. a control group.

## Data Availability

The data used to support the findings of this study are available from the corresponding author upon request.
